The article "Molecular characterization of Legionella pneumophila-induced interleukin-8 expression in T cells" was retracted in 2011. Reason: duplicated images.

# Molecular characterization of *Legionella pneumophila*-induced interleukin-8 expression in T cells

**DOI:** 10.1186/1471-2180-10-1

**Published:** 2010-01-05

**Authors:** Reika Takamatsu, Hiromitsu Teruya, Eriko Takeshima, Chie Ishikawa, Kunihiro Matsumoto, Naofumi Mukaida, Jian-Dong Li, Klaus Heuner, Futoshi Higa, Jiro Fujita, Naoki Mori

**Affiliations:** 1 Division of Molecular Virology and Oncology, Graduate School of Medicine, University of the Ryukyus, 207 Uehara, Nishihara, Okinawa 903-0215, Japan; 2 Division of Control and Prevention of Infectious Diseases, Graduate School of Medicine, University of the Ryukyus, 207 Uehara, Nishihara, Okinawa 903-0215, Japan; 3 Transdisciplinary Research Organization for Subtropics and Island Studies, University of the Ryukyus, 1 Senbaru, Nishihara, Okinawa 903-0215, Japan; 4 Department of Molecular Biology, Graduate School of Science, Nagoya University, Chikusa-ku, Nagoya 464-8602, Japan; 5 Division of Molecular Bioregulation, Cancer Research Institute, Kanazawa University, 13-1 Takara-machi, Kanazawa 920-0934, Japan; 6 Department of Microbiology and Immunology, University of Rochester Medical Center, 601 Elmwood Avenue, Rochester, New York 14642, USA; 7 Project group 26 "Nosocomial Infections of the Elderly", Robert Koch-Institut, 20 Nordufer, Berlin 13353, Germany

## Abstract

**Background:**

*Legionella pneumophila *is the causative agent of human Legionnaire's disease. During infection, the bacterium invades macrophages and lung epithelial cells, and replicates intracellularly. However, little is known about its interaction with T cells. We investigated the ability of *L. pneumophila *to infect and stimulate the production of interleukin-8 (IL-8) in T cells. The objective of this study was to assess whether *L. pneumophila *interferes with the immune system by interacting and infecting T cells.

**Results:**

Wild-type *L. pneumophila *and flagellin-deficient *Legionella*, but not *L. pneumophila *lacking a functional type IV secretion system Dot/Icm, replicated in T cells. On the other hand, wild-type *L. pneumophila *and Dot/Icm-deficient *Legionella*, but not flagellin-deficient *Legionella *or heat-killed *Legionella *induced IL-8 expression. *L. pneumophila *activated an IL-8 promoter through the NF-κB and AP-1 binding regions. Wild-type *L. pneumophila *but not flagellin-deficient *Legionella *activated NF-κB, p38 mitogen-activated protein kinase (MAPK), Jun N-terminal kinase (JNK), and transforming growth factor β-associated kinase 1 (TAK1). Transfection of dominant negative mutants of IκBα, IκB kinase, NF-κB-inducing kinase, TAK1, MyD88, and p38 MAPK inhibited *L. pneumophila*-induced IL-8 activation. Inhibitors of NF-κB, p38 MAPK, and JNK blocked *L. pneumophila*-induced IL-8 expression. In addition, c-Jun, JunD, cyclic AMP response element binding protein, and activating transcription factor 1, which are substrates of p38 MAPK and JNK, bound to the AP-1 site of the IL-8 promoter.

**Conclusions:**

Taken together, *L. pneumophila *induced a flagellin-dependent activation of TAK1, p38 MAPK, and JNK, as well as NF-κB and AP-1, which resulted in IL-8 production in human T cells, presumably contributing to the immune response in Legionnaire's disease.

## Background

The gram-negative bacteria *Legionella pneumophila *is the causative pathogen of Legionnaires' disease, a potentially fatal type of pneumonia affecting both immunocompromised and immunocompetent subjects. This bacterium is a facultative intracellular pathogen of amoeba in natural and man-made aquatic environments. Infection of humans occurs after inhalation of contaminated water aerosol droplets. Dependent on its type IV secretion system Dot/Icm, *L. pneumophila *initiates biogenesis of a specialized vacuole that it critical for *Legionella *replication [1]. This *Legionella*-containing vacuole avoids fusion with lysosomes and acquires vesicles from the endoplasmic reticulum [2]. In addition, the bacterial flagellum with its major component flagellin is also considered to represent a virulence-associated factor [3].

For *L. pneumophila *pathogenesis, important results were obtained by analyzing infection of protozoans or immune cells like macrophages [4]. However, recent studies have shown that *L. pneumophila *replicates also in human alveolar epithelial cells [5,6]. Although *Legionella *less efficiently replicates within human T cells compared with macrophages [7], little is known of the consequences of T cell infection with *Legionella*.

The objective of this study was to assess whether *L. pneumophila *interferes with the immune system by interacting and infecting T cells. The results demonstrated that *L. pneumophila *interacted with and infected T cells. To investigate *L. pneumophila*-T cell interactions, we examined whether *L. pneumophila *induces production of interleukin-8 (IL-8), an inflammatory chemokine associated with immune-mediated pathology and involved in recruitment and activation of neutrophils and other immune cells. The results showed that *L. pneumophila *directly increased IL-8 by activation of transforming growth factor β-associated kinase 1 (TAK1), p38 mitogen-activated protein kinase (MAPK), and Jun N-terminal kinase (JNK), leading to activation of transcription factors, NF-κB, AP-1, cyclic AMP response element (CRE) binding protein (CREB), and activating transcription factor-1 (ATF1).

## Results

### Multiplication of *L. pneumophila *in human T cells

To investigate the interaction of *L. pneumophila *with T cells, we first examined intracellular growth of *L. pneumophila *strain AA100jm in Jurkat cells by 72-h continuous cultures. The CFU per well of AA100jm growing in Jurkat cell cultures began to increase after 24 h and then increased time-dependently (Fig. 1A). However, the CFU of the avirulent mutant strain with a knockout in *dotO*, encoding a protein essential for type IV secretion system, did not increase during the 72-h period (Fig. 1A). In contrast, the multiplication of *flaA *mutant did not change in Jurkat cells compared with the wild-type Corby (Fig. 1B). To characterize the multiplication of *L. pneumophila *in human T cells, intracellular growth in CD4^+ ^T cells of *L. pneumophila *was examined. The CFU of the wild-type Corby increased after infection for 24 h in CD4^+ ^T cells, although it replicated less efficiently compared with the observations with Jurkat cells (Fig. 1C). Staining of the infected Jurkat cells for *L. pneumophila *showed increased intracellular replication of AA100jm, Corby, and *flaA *mutant, but not *dotO *mutant after 24 h in culture (Fig. 1D and 1E). These observations suggest that *L. pneumophila *can replicate in human T cells and the type IV secretion system plays a role in *L. pneumophila *replication in human T cells.

**Figure 1:** **Intracellular growth of *L. pneumophila *strains in Jurkat cells and CD4^+ ^T cells**. Jurkat cells were infected with *L. pneumophila *strains AA100jm and *dotO *mutant (MOI of 100) (A) or Corby and *flaA *mutant (MOI of 100) (B). (C) CD4^+ ^T cells were also infected with Corby (MOI of 50). At the indicated time points after infection, the CFU was enumerated. Data are mean ± SD of triplicate cell cultures. (D and E) Direct fluorescent antibody staining of *L. pneumophila *strains. Jurkat cells were infected with AA100jm and *dotO *mutant (MOI of 100) (D) or Corby and *flaA *mutant (MOI of 100) (E) for 24 h. Jurkat cells were stained with fluorescein-conjugated anti-*L. pneumophila *antibody. Original magnification, ×600.

### High serum IL-8 levels in patients with *Legionella *pneumonia

To investigate the role of IL-8 in the pathogenesis of *Legionella *pneumonia, the circulating concentrations of IL-8 were measured. Serum IL-8 levels were higher in patients with *Legionella *pneumonia (*n *= 18) (189 ± 493 pg/ml) than in normal healthy controls (*n *= 16) (9.79 ± 15.06 pg/ml), although this difference was not statistically significant (*P *= 0.157). Therefore, we analyzed the signaling pathways for IL-8 activation by *Legionalla *infection.

### Infection of Jurkat and CD4^+ ^T cells by *L. pneumophila *induces IL-8 expression

Jurkat cells were infected with wild-type *L. pneumophila *strains AA100jm and Corby for up to 12 h. Total cellular RNA was isolated from these cells at 0.5, 1, 2, 4, 6, 8 and 12 h after the infection and IL-8 gene expression was analyzed by RT-PCR. IL-8 mRNA expression increased after the infection (Fig. 2A). In another series of experiments, in which Jurkat cells were infected with AA100jm and Corby at different concentrations for 4 h (Fig. 2B), both strains induced dose-dependent expression of IL-8 mRNA. Next, we examined the correlation between IL-8 expression levels and the virulence of *L. pneumophila*. As shown in Fig. 2A, IL-8 mRNA expression was induced after infection with the avirulent *dotO *mutant, but became gradually weaker from 8 to 12 h. In contrast, a *flaA *knockout mutant, defective in flagellin production, failed to induce IL-8 mRNA after infection (Fig. 2A). To characterize the effect of *L. pneumophila *infection on human T cells, IL-8 mRNA expression in CD4^+ ^T cells in response to *L. pneumophila *was examined by RT-PCR. After infection for 3 h, *L. pneumophila *induced IL-8 mRNA expression in CD4^+ ^T cells, similar to the observations with Jurkat cells (Fig. 2C).

**Figure 2:** ***L. pneumophila*-induced IL-8 mRNA expression in T cells**. (A) Total RNA was extracted from Jurkat cells infected with AA100jm, *dotO *mutant, Corby, or *flaA *mutant (MOI of 100) for the indicated time intervals and used for RT-PCR. (B) Jurkat cells were infected with the indicated concentrations of *L. pneumophila *for 4 h. Total RNA was extracted and used for RT-PCR. (C) Total RNA was extracted from CD4^+ ^T cells infected with Corby (MOI of 50) for 3 h and used for RT-PCR. (D) Jurkat cells were infected with live *L. pneumophila *Corby or *flaA *mutant (MOI of 100) for 4 h or incubated with *L. pneumophila *under the indicated treatment for 4 h. PFA, paraformaldehyde. Total RNA was extracted and used for RT-PCR. Representative examples of three experiments with similar results.

To determine the correlation between IL-8 expression level and *L. pneumophila *bacterial proteins, heat-killed Corby was used to infect Jurkat cells at a multiplicity of infection (MOI) of 100. At 4 h, IL-8 was not expressed in Jurkat cells infected with the heat-killed strain (Fig. 2D). Furthermore, IL-8 gene expression was not induced when paraformaldehyde-fixed *L. pneumophila *was used (Fig. 2D). However, bacteria heated at 56°C for 30 min induced IL-8 expression. These results suggest that the surface proteins of bacteria but not lipopolysaccharide are required for IL-8 induction. Considered together, it seems that *Legionella *flagellin is involved in IL-8 expression in T cells.

Flagellin is recognized by toll-like receptor 5 (TLR5) [8]. Thus, we also examined the expression of TLR2, TLR3, TLR4, and TLR5 mRNAs in Jurkat and CD4^+ ^T cells. All TLR mRNAs examined were expressed in Jurkat and CD4^+ ^T cells (Fig. 3A and 3B). Furthermore, their expression levels did not change by *L. pneumophila *infection in CD4^+ ^T cells (Fig. 3B) and Jurkat cells (data not shown).

**Figure 3:** **TLR mRNA expression in T cells**. (A) Expression of TLR mRNA in Jurkat cells. Total RNA was extracted from Jurkat cells and used for RT-PCR. (B) CD4^+ ^T cells were infected without or with Corby (MOI of 50) for 3 h. Total RNA was extracted from CD4^+ ^T cells and used for RT-PCR. Representative examples of three experiments with similar results.

### IL-8 production from Jurkat cells during infection with *L. pneumophila*

We used enzyme-linked immunosorbent assay (ELISA) to determine IL-8 protein levels in culture supernatants of Jurkat cells at 8, 12, or 24 h after infection with either the parental strain Corby or *flaA *mutant strain at an MOI of 100. IL-8 was induced by Corby in a time-dependent manner. On the other hand, the amount of IL-8 produced by Jurkat cells infected with the *flaA *mutant strain was significantly less than that by cells infected with the wild-type strain (Fig. 4A). Corby-induced IL-8 production by Jurkat cells was MOI-dependent (Fig. 4B). Corby also induced a significant amount of IL-8 from CD4^+ ^T cells (Fig. 4C).

**Figure 4:** **IL-8 production from Jurkat cells during infection with *L. pneumophila *strains**. (A) Jurkat cells were infected with the indicated *L. pneumophila *strains at an MOI of 100 for the indicated time periods. (B) Jurkat cells were infected with the varying concentrations of the indicated *L. pneumophila *strains for 24 h. (C) CD4^+ ^T cells were infected without or with Corby for 3 h. IL-8 concentrations in the supernatants were determined by ELISA. Data are mean ± SD values collected in three experiments.

### *L. pneumophila *induces IL-8 gene transcription via a sequence spanning positions -133 to -50 of the IL-8 gene promoter

To delineate the mechanism by which *L. pneumophila *induces IL-8 gene transcription, we identified *L. pneumophila*-responsive promoter elements in the IL-8 promoter. This was achieved by transfecting Jurkat cells with various plasmid constructs containing the luciferase reporter gene driven by the IL-8 promoter. Twenty-four hours post-transfection, cells were infected with *L. pneumophila *strain Corby. *L. pneumophila *infection resulted in activation of the 5' region 1,481 bp full-length promoter in an MOI-dependent manner (Fig. 5A). These results indicate that *L. pneumophila *induces IL-8 expression in Jurkat cells at transcriptional level. Next, we used a deletion analysis approach to identify the essential promoter element(s) for transcriptional upregulation following a stimulus. High induction levels were observed with a reporter construct containing IL-8 5'-flanking sequence starting with position -1,481 to position -133. Deletion of sequences upstream of position -50 abolished induction of IL-8 by *L. pneumophila *infection (Fig. 5B). The IL-8 gene fragment spanning positions -133 to -50 bp contains three prominent DNA-protein interaction sites for the transcription factors AP-1, nuclear factor IL-6 (NF-IL-6), and NF-κB (Fig. 5B). This maps the region from -133 to -50 bp as a *L. pneumophila*-responsive region, which is likely to contain individual *L. pneumophila*-responsive regulatory elements.

**Figure 5:** ***L. pneumophila *infection activates IL-8 promoter in Jurkat cells**. (A) Jurkat cells transfected with -1481-luc were infected with *L. pneumophila *Corby at the indicated MOI values for 6 h. The luciferase activities were expressed relative to cells transfected with -1481-luc followed by mock-infection. *, *P *< 0.01, as determined by the Student *t *test. (B) Reporter assay using plasmid DNA containing serial deletions in 5'-flanking region of the IL-8 gene. (Left) Schematic representation of the IL-8 reporter constructs, demonstrating locations of several known binding sites for transcription factors. (Right) The indicated luciferase reporter constructs were transfected into Jurkat cells, and the cells were subsequently infected with Corby strain (MOI of 100) for 6 h. The activities are expressed relative to that of cells transfected with -50-luc followed by mock-infection, which was defined as 1. The numbers on the bars depict fold induction relative to the basal level measured in uninfected cells. (C) Relative importance of AP-1, NF-IL-6, and NF-κB binding sites in IL-8 promoter. Wild-type and mutated plasmids were transfected into Jurkat cells. The transfected cells were infected without or with Corby. The activities are expressed relative to that of cells transfected with -133-luc followed by mock-infection, which was defined as 1. Luciferase activities were normalized based on the *Renilla *luciferase activity from phRL-TK. The numbers on the bars depict fold induction relative to the basal level measured in uninfected cells. LUC, luciferase. Graph data are mean ± SD values of three experiments.

To identify the *cis*-acting element(s) in the -133 to -50 bp region of the IL-8 promoter, which served as a *L. pneumophila*-responsive regulatory element, we prepared and tested site-directed mutant constructs (Fig. 5C). Mutation in the NF-κB site (NF-κB mut-luc) and AP-1 site (AP-1 mut-luc) suppressed *L. pneumophila*-induced IL-8 expression. However, mutation of the NF-IL-6 site (NF-IL-6 mut-luc) had no such effect. These results indicate that activation of the IL-8 promoter in Jurkat cells in response to *L. pneumophila *infection requires an intact binding site for the NF-κB and AP-1 elements.

### Flagellin-dependent activation of NF-κB

Because the internal mutational analysis of IL-8 promoter indicated that *L. pneumophila *infection activated transcription through the NF-κB site, it was important to identify the nuclear factor(s) that binds to this site. The NF-κB sequence derived from the IL-8 promoter was used as a probe in electrophoretic mobility shift assay (EMSA). Jurkat cells were infected with Corby strain at different times after challenge, and nuclear protein extracts were prepared and analyzed to determine NF-κB DNA binding activity. As shown in Fig. 6A, a complex was induced in these cells within 30 min after infection with Corby and increased in a time-dependent manner. This NF-κB binding activity to IL-8 promoter was reduced by the addition of either cold probe or a typical NF-κB sequence derived from the IL-2 receptor (IL-2R) α-chain (IL-2Rα) enhancer but not by an oligonucleotide containing the AP-1 binding site (Fig. 6B, lanes 3 to 5). Next, we characterized the *L. pneumophila*-induced complexes identified by the IL-8 NF-κB probe. These complexes were diminished and supershifted by the addition of anti-p50 or anti-p65 antibody (Fig. 6A, lanes 6 to 10), suggesting that *L. pneumophila*-induced IL-8 NF-κB complexes are composed of p50 and p65. Based on these results, one can conclude that *L. pneumophila *infection seems to induce IL-8 gene expression at least in part through induced binding of p50 and p65 to the NF-κB site in the IL-8 promoter region.

**Figure 6:** **NF-κB signal is essential for flagellin-dependent activation of the IL-8 promoter by *L. pneumophila***. (A) Flagellin is required for induction of NF-κB binding activity. Nuclear extracts from Jurkat cells infected with Corby or *flaA *mutant were mixed with IL-8 NF-κB probe (MOI, 100:1). (B) Sequence specificity of NF-κB binding activity and characterization of proteins that bound to the NF-κB binding site. Competition assays were performed with nuclear extracts from cells infected with Corby for 2 h. 100-fold excess amounts of competitor were added (lanes 3 to 5). A supershift assay in the same nuclear extracts also was performed. Antibodies (Ab) were added (lanes 6 to 10). Arrows indicate specific complexes, while arrowheads indicate the DNA binding complexes supershifted. (C) Flagellin-induced p65 translocation. Cells were infected with Corby or *flaA *mutant. Nuclear extracts were subjected to immunoblotting. (D) Flagellin activates NF-κB through the classical and alternative pathways. Cells were infected with Corby or *flaA *mutant. Lysates were subjected to immunoblotting. (E) Overexpression of dominant negative mutants inhibits *L. pneumophila*-induced activation of the IL-8 promoter. Cells were transfected with -133-luc and the mutant plasmids and then infected with Corby for 6 h. The solid bar indicates luciferase activity of -133-luc and empty vector without infection. Activity is expressed relative to that of cells transfected with -133-luc with further Corby infection, which was defined as 100. Data are means ± SD values of three experiments. dn, dominant negative. *, *P *< 0.05; **, *P *< 0.001 (by Student *t *test).

As described above, the *flaA *mutant strain failed to induce mRNA expression and production of IL-8. Next, we determined whether the *flaA *mutant strain induces NF-κB DNA binding activity. As expected, NF-κB DNA binding activity was not induced by the isogenic *flaA *mutant, unlike the wild-type strain Corby (Fig. 6A). These results indicate that better activation of NF-κB binding by *flaA*-positive strain is the underlying mechanism of the observed activation of the IL-8 promoter by this bacterial strain. Considered together, these results indicate that *L. pneumophila *infection induces IL-8 gene expression at least in part through the induced binding of p50 and p65 NF-κB family members to the NF-κB element of the IL-8 promoter and that this effect is dependent on flagellin.

Because nuclear translocation is a key step for transcriptional activity [9], we next examined whether *L. pneumophila *induces the nuclear translocation of NF-κB. As shown in Fig. 6C, the wild-type Corby, but not the *flaA *mutant, induced nuclear translocation of NF-κB. NF-κB is normally present in the cytoplasm in an inactive state and is bound to members of the IκB inhibitor protein family, chiefly IκBα. In this complex, IκBα blocks the nuclear localization signal, thus preventing nuclear translocation. Translocation of NF-κB into the nucleus requires disruption of the cytoplasmic NF-κB:IκBα complex [9]. To determine the role of IκBα phosphorylation and degradation in *L. pneumophila*-induced NF-κB translocation and activation, we investigated whether *L. pneumophila *induces phosphorylation and degradation of IκBα. The latter two processes were examined by Western blot analysis using antibodies against phosphorylated and total IκBα, respectively. Fig. 6D shows phosphorylation and degradation of IκBα in Jurkat cells infected with the wild-type Corby but not the *flaA *mutant for 1, 2 and 4 h. The IκBα phosphorylation became evident at 1 h and decreased thereafter. Consistent with this, Corby-induced degradation of IκBα was observed at 1 h.

NF-κB signaling occurs either through the classical or alternative pathway [10]. In the classical pathway, NF-κB dimers, such as p50/p65, are maintained in the cytoplasm by interaction with IκBα. Whereas the classical NF-κB activation is IκB kinase β(IKKβ)- and IKKγ-dependent and occurs through IκBα phosphorylation and subsequent proteasomal degradation, the alternative pathway depends on IKKα homodimers and NF-κB-inducing kinase (NIK) and results in regulated processing of the p100 precursor protein to p52 via phosphorylation and degradation of its IκB-terminus [10]. Indeed, the wild-type Corby but not the *flaA *mutant induced phosphorylation of p65 and upstream kinase IKKβ (Fig. 6D). Next, we examined the alternative pathway, which involves the cleavage of NF-κB2/p100 to p52. The level of p52 protein increased in Jurkat cells infected with the wild-type Corby but not the *flaA *mutant (Fig. 6D), indicating that flagellin activates NF-κB via the alternative pathway.

### NF-κB signal is essential for induction of IL-8 expression by *L. pneumophila*

To further confirm the involvement of IκBα degradation, we transfected the cells with transdominant mutant of IκBα in which two critical serine residues required for inducer-mediated phosphorylation were deleted [11]. As seen in Fig. 6E, overexpression of mutant IκBα greatly inhibited the Corby-induced IL-8 promoter activation. This observation implicates the involvement of IκBα phosphorylation and degradation in flagellin-induced IL-8 expression.

To address the mechanism of flagellin-mediated IL-8 expression, we investigated the role of NIK and IKK in *L. pneumophila*-induced IL-8 expression. Cotransfection with the dominant-negative mutant forms of NIK, IKKα, IKKβ, and IKKγ inhibited *L. pneumophila*-induced IL-8 expression (Fig. 6E). MyD88 is a universal adaptor for induction of cytokines by TLR2, TLR4, TLR5, TLR7, and TLR9. It is also required for activation of NF-κB by these TLRs [12]. Likewise, overexpression of a dominant negative mutant form of MyD88 also inhibited *L. pneumophila*-induced IL-8 expression. Taken together, these findings clearly demonstrate that *L. pneumophila *induces IL-8 expression via activation of flagellin-dependent NF-κB signaling pathway.

Because activation of the IL-8 promoter by *L. pneumophila *infection required the activation of NF-κB, we blocked NF-κB activation with Bay 11-7082, an inhibitor of IκBα phosphorylation [13]. Bay 11-7082 markedly inhibited *L. pneumophila*-induced phosphorylation and degradation of IκBα, as well as NF-κB DNA binding (Fig. 7A and 7B). Furthermore, Bay 11-7082 resulted in a dose-dependent reduction in *L. pneumophila*-induced IL-8 mRNA expression and secretion by Jurkat cells (Fig. 7C and 7D).

**Figure 7:** **Bay 11-7082 blocks *L. pneumophila*-induced NF-κB activation and IL-8 secretion**. Jurkat cells were pretreated with or without Bay 11-7082 (20 μM) for 1 h prior to *L. pneumophila *Corby infection and subsequently were infected with Corby (MOI, 100:1) for the indicated times. Cell lysates were prepared and subjected to immunoblotting with the indicated antibodies (A) and nuclear extracts from the harvested cells were analyzed for NF-κB and Oct-1 (B). Jurkat cells were pretreated with the indicated concentrations of Bay 11-7082 for 1 h prior to Corby infection and subsequently infected with Corby (MOI, 100:1) for 4 h (C) and 24 h (D). IL-8 mRNA expression on the harvested cells was analyzed by RT-PCR (C) and the supernatants were subjected to ELISA to determine IL-8 secretion (D). Data in (A)-(C) are representative examples of three independent experiments with similar results. Data are mean ± SD from three experiments.

### Flagellin-dependent activation of AP-1

To obtain further evidence for the AP-1 site on the IL-8 promoter in response to *L. pneumophila*, we examined the nuclear factors that bind to this site. The AP-1 sequence derived from the IL-8 promoter was used as a probe in EMSA. Jurkat cells were infected with the wild-type Corby or the *flaA *mutant at different times after challenge, and nuclear protein extracts were prepared and analyzed to determine AP-1 DNA binding activity. As shown in Fig. 8A, markedly increased complexes were induced by Corby compared with that induced by the isogenic *flaA *mutant. These results indicate that better activation of AP-1 binding by the flagellin-positive strain is the underlying mechanism of the observed activation of the IL-8 promoter by *L. pneumophila*. This AP-1 binding activity to the IL-8 promoter was reduced by the addition of either cold probe or a CREB sequence but not by an NF-κB sequence derived from the IL-2Rα enhancer (Fig. 8B, lanes 2 to 4).

**Figure 8:** ***L. pneumophila *activates AP-1 signal through flagellin**. (A) Time course of AP-1 activation in Jurkat cells infected with *L. pneumophila*, evaluated by EMSA. Nuclear extracts from Jurkat cells, infected with Corby or *flaA *mutant (MOI, 100:1), for the indicated time periods, were mixed with IL-8 AP-1 ^32^P-labeled probe. (B) Sequence specificity of AP-1 binding activity and characterization of AP-1/CREB/ATF proteins that bound to the AP-1 binding site of the IL-8 gene. Competition assays were performed with nuclear extracts from Jurkat cells infected with Corby for 2 h. Where indicated, 100-fold excess amounts of each specific competitor oligonucleotide were added to the reaction mixture with labeled probe AP-1 (lanes 2 to 4). A supershift assay of AP-1 DNA binding complexes in the same nuclear extracts also was performed. Where indicated, appropriate antibodies (Ab) were added to the reaction mixture before the addition of the ^32^P-labeled probe (lanes 6 to 17 and 19). Arrows indicate specific complexes, while arrowheads indicate the DNA binding complexes supershifted by antibodies. (C) Jurkat cells were infected with Corby or *flaA *mutant for the indicated time periods. Cell lysates were prepared and subjected to immunoblotting with the indicated antibodies. Data are representative examples of three independent experiments with similar results.

Next, we characterized the *L. pneumophila*-induced complexes identified by the IL-8 AP-1 probe. These complexes were diminished and supershifted by the addition of anti-c-Jun, anti-JunD, anti-ATF1, or anti-CREB antibody (Fig. 8B, lanes 10, 12, 13, and 17). The addition of these four antibodies completely diminished AP-1 DNA binding (Fig. 8B, lane 19). These results suggest that flagellin-induced IL-8 AP-1 complexes are composed of c-Jun, JunD, ATF1, and CREB to the AP-1 site in the IL-8 promoter region. Next, we examined phosphorylation of these four proteins in Jurkat cells infected with Corby or the isogenic *flaA *mutant. Corby but not *flaA *mutant enhanced phosphorylation of c-Jun, JunD, ATF1, and CREB in a time-dependent manner (Fig. 8C). These transcription factors are phosphorylated by p38 MAPK, JNK, and extracellular signal-regulated kinase (ERK) [14-18]. Furthermore, activated MAPKs phosphorylate AP-1, CREB, and ATF complexes, which results in increased AP-1-dependent transcription. We investigated whether *L. pneumophila *Corby activates these MAPKs.

### The p38 MAPK pathway mediates activation of CREB and ATF1 by flagellin

Phosphorylation of p38 MAPK by Corby was determined by Western blot analysis (Fig. 9A). Corby, but not the *flaA *mutant, phosphorylated MAPKAPK-2 and MSK1, downstream CREB/ATF kinases of p38 MAPK in Jurkat cells (Fig. 9A). Consistent with the role of p38 MAPK phosphorylation in Jurkat cells infected with Corby in IL-8 expression and release, SB203580, a p38 MAPK inhibitor, reduced Corby-induced IL-8 expression and release by Jurkat cells in a dose-dependent manner (Fig. 9B and 9C). Furthermore, SB203580 inhibited Corby-induced luciferase activity of the IL-8 promoter in a dose-dependent manner (Fig. 9D). Similarly, overexpression of a dominant-negative mutant form of either p38α or p38β also inhibited Corby-induced luciferase activity of the IL-8 promoter, confirming the involvement of p38 MAPK in flagellin-induced IL-8 expression (Fig. 9E). The finding that SB203580 prevented Corby-induced phosphorylation of CREB and ATF1, and MAPKAPK-2 and MSK1, downstream targets of p38 MAPK (Fig. 9F), suggests that MAPKAPK-2 and MSK1 seem to mediate the flagellin-induced phosphorylation of CREB and ATF1.

**Figure 9:** **MAPKs activation by *L. pneumophila *through flagellin and inhibition of *L. pneumophila*-induced CREB and ATF1 activation and IL-8 transcription by p38 inhibitor**. (A) Jurkat cells were infected with Corby or *flaA *mutant (MOI, 100:1), and lysates were subjected to immunoblotting. Cells were pretreated with the indicated concentrations of SB203580 for 1 h prior to infection and subsequently infected with Corby (MOI, 100:1) for 4 h (B) and for 6, 8, 12, or 24 h (C). IL-8 mRNA expression on the harvested cells was analyzed by RT-PCR (B) and the supernatants were subjected to ELISA to determine IL-8 secretion (C). (D) Cells were transfected with -133-luc and then pretreated with the indicated concentrations of SB203580 for 1 h prior to infection. They were infected subsequently with Corby for 6 h. Luciferase (LUC) activity was assayed. The solid bar indicates LUC activity of -133-luc without infection. (E) Cells were transfected with -133-luc and dominant negative mutants and then infected with Corby for 6 h. The solid bar indicates LUC activity of -133-luc without infection. All values were calculated as the change (*n*-fold) in induction values relative to the basal level measured in uninfected cells. Data are mean ± SD of three experiments. (F) Cells were pretreated with or without SB203580 (50 μM) for 1 h prior to infection and subsequently were infected with Corby (MOI, 100:1). Lysates were subjected to immunoblotting. dn, dominant negative.

### Effects of JNK and ERK on flagellin-induced IL-8 expression

We also examined the effect of flagellin on activation of JNK and ERK. Corby, but not the *flaA *mutant, markedly increased the phosphorylation of JNK and MAPK kinase 4 (MKK4), upstream activator of JNK, and ERK in Jurkat cells (Fig. 9A). In addition, SP600125, an inhibitor of JNK, suppressed Corby-induced IL-8 expression and release in a dose-dependent manner (Fig. 10A and 10B). The finding that SP600125 inhibited Corby-induced phosphorylation of c-Jun but not JunD (Fig. 10C), suggests that JNK seems to mediate the flagellin-induced phosphorylation of c-Jun.

**Figure 10:** **SP600125 inhibits *L. pneumophila*-induced IL-8 expression and secretion**. Jurkat cells were pretreated with the indicated concentrations of SP600125 for 1 h prior to *L. pneumophila *Corby infection and subsequently infected with Corby (MOI, 100:1) for 4 h (A) and 24 h (B). IL-8 mRNA expression on harvested cells was analyzed by RT-PCR (A) and the supernatants were subjected to ELISA to determine IL-8 secretion (B). Data are mean ± SD of three experiments. (C) Jurkat cells were pretreated with or without SP600125 (20 μM) for 1 h prior to *L. pneumophila *Corby infection and subsequently infected with Corby (MOI, 100:1) for the indicated times. Cell lysates were prepared and subjected to immunoblotting with the indicated antibodies. Data in (A) and (C) are representative examples of three independent experiments with similar results.

To determine the direct role of ERK phosphorylation in *L. pneumophila*-induced IL-8 expression, Jurkat cells were infected with Corby in the absence or presence of PD98059, an inhibitor of MEK1/2, an upstream activator of ERK. RNA and supernatants were collected after 4 and 24 h of infection and assayed for IL-8 mRNA expression and release, respectively. The addition of PD98059 had no effect on *L. pneumophila*-induced IL-8 mRNA expression and release by Jurkat cells (Fig. 11A and 11B). The activity of this inhibitor was verified by examining the phosphorylation state of ERK in *L. pneumophila*-infected cells after selected incubation time periods with PD98059. Whereas ERK activity was reduced in Jurkat cells in the presence of the inhibitor, the phosphorylation of CREB, ATF1, c-Jun, and JunD was not affected (Fig. 11C).

**Figure 11:** **TAK1 but not ERK plays key roles in *L. pneumophila*-induced IL-8 expression**. (A) Jurkat cells were pretreated with the indicated concentrations of PD98059 for 1 h prior to *L. pneumophila *Corby infection and subsequently infected with Corby (MOI, 100:1) for 4 h (A) and 24 h (B). IL-8 mRNA expression on harvested cells was analyzed by RT-PCR (A) and the supernatants were subjected to ELISA to determine IL-8 secretion (B). Data are mean ± SD of three experiments. (C) Jurkat cells were pretreated with or without PD98059 (50 μM) for 1 h prior to *L. pneumophila *Corby infection and subsequently infected with Corby (MOI, 100:1) for the indicated times. Cell lysates were prepared and subjected to immunoblotting with the indicated antibodies. (D) Jurkat cells were transfected with -133-luc and a dominant negative mutant of TAK1 or empty vector and then infected with Corby for 6 h. The solid bar indicates LUC activity of -133-luc without Corby infection. The activities are expressed relative to that of cells transfected with -133-luc and empty vector without further Corby infection, which was defined as 1. Data are mean ± SD of three experiments. Data in (A) and (C) are representative examples of three independent experiments with similar results.

### Effect of TAK1 on flagellin-induced IL-8 expression

TAK1 is one of the most characterized MAPK kinase kinase family members and is activated by various cellular stresses including IL-1 [19,20]. TAK1 functions as an upstream stimulatory molecule of the JNK, p38 MAPK, and IKK signaling pathways. Accordingly, we investigated whether TAK1 is also involved in *L. pneumophila*-induced IL-8 expression. As shown in Fig. 9A, phosphorylation of TAK1 was induced in Jurkat cells infected with Corby but not with *flaA *mutant. Furthermore, a dominant negative mutant of TAK1 inhibited *L. pneumophila*-induced IL-8 activation (Fig. 11D). These data suggest that trifurcation of *L. pneumophila *flagellin-induced IKK-IκB, MKK4-JNK, and p38 MAPK signaling pathways occurs at TAK1.

## Discussion

Innate immunity is essential for limiting *L. pneumophila *infection at cellular and microbe levels. TLRs are involved in controlling *L. pneumophila *infection *in vivo*, since mice lacking TLR2 are more susceptible to infection, and MyD88-deficient mice show defective control of *L. pneumophila *infection [21,22]. Knowledge about host immunoreaction against *L pneumophila *is mainly based on studies on macrophages. While adaptive immunity has been shown to be important for host resistance to *L. pneumophila *[23], the direct interaction of bacteria with adaptive immune cells such as T cells is not well known. In this study, we show that *L. pneumophila *stimulates Jurkat T cells. Furthermore, this stimulation of T cells is mainly provided by flagellin since the *flaA *mutant was deficient in stimulating T cells to produce IL-8. This difference was independent of bacterial replication, as the *flaA *mutant could replicate in Jurkat T cells. Although *Legionella *less efficiently replicates within T cells, it is possible that uninfected T cells might respond to extracellular flagellin. Whether or not T cells are infected with *L. pneumophila in vivo*, they might still conceivably be a source of IL-8, because extracellular flagellin could induce IL-8 expression [24] and induction of IL-8 by *L. pneumophilla *did not require invasion. Interestingly, TLR5-deficient mice had lower numbers of polymorphonuclear neutrophils in their broncho-alveolar lavage fluid in comparison to wild-type mice after *Legionella *infection [25].

Infection with flagellin-deficient *L. pneumophila *has been reported to induce a robust cytokine response equivalent to infection with wild-type *L. pneumophila *in macrophages [26]. This cytokine response requires a functional *L. pneumophila *Dot/Icm type IV secretion system in macrophages and dendritic cells [26-28], indicating that T cells are unique. Although bacterial lipoprotein can also stimulate T cells [29,30], stimulation with lipoprotein of *L. pneumophila *has not yet been shown for human T cells.

In this study, we demonstrated that *L. pneumophila *induces IL-8 expression through flagellin and NF-κB signaling pathway modulates this induction in human T cells. Using a specific pharmacological inhibitor, we showed that IKK-NF-κB pathway augmented *L. pneumophila *induction of IL-8 expression. We confirmed the important role of NF-κB by showing that overexpression of dominant negative NIK, IKKs, and IκBα, potent inhibitors of NF-κB activation, inhibited IL-8 promoter activation by *L. pneumophila*. The alternative pathway proceeds via NIK-, IKKα, and protein synthesis-dependent processing of the p100 precursor protein to the p52 form and resulted in a delayed but sustained activation of primarily RelB-containing NF-κB dimmers [10]. The *Legionella *type IV effector LegK1 has been recently reported to process p100 into p52 [31]. The dominant negative mutants of NIK and IKKα inhibited IL-8 promoter activation by *L. pneumophila *in Jurkat cells. Furthermore, *L. pneumophila *infection induced p100 processing into p52 subunit, although supershift experiments did not reveal that the NF-κB-DNA binding complexes in Jurkat cells infected with *L. pneumophila *involve p52 and RelB. Further basic investigations with knockout and knockdown experiments will be essential in exploring the involvement of NIK-dependent alternative NF-κB pathway in *L. pneumophila *flagellin-induced IL-8 expression in T cells.

Recently, infection with *L. pneumophila *has been shown to induce a biphasic activation of NF-κB in human epithelial cells: (i) early in infection, bacterial flagellin induces signaling of TLR5 and a transient translocation of p65 into the nucleus and (ii) at later time points, an unknown factor that depends on bacterial replication and a functional Dot/Icm system induces continuous nuclear localization of p65 and permanent degradation of IκBα [32]. Certainly, IL-8 mRNA expression was induced immediately after the infection, but became gradually weaker from 8 to 12 h after infection with the *dotO *mutant in Jurkat cells. *L. pneumophila *could also induce biphasic activation of NF-κB in T cells. The Dot/Icm system was demonstrated to be necessary for NF-κB activation in infections of human macrophages [33,34]. Furthermore, the Corby strain was shown to have a severely reduced Dot/Icm-dependent NF-κB activation [32]. Therefore, the *flaA *mutant derived from Corby strain might be deficient in infecting T cells to produce IL-8. In addition to flagellin, the Dot/Icm system might also be necessary for NF-κB activation and subsequent upregulation of IL-8 gene in infections of T cells.

In addition to NF-κB activation, MAPKs have also been implicated in the induction of IL-8 production [35]. The data presented here showing that all three MAPKs (p38, JNK, and ERK) were consistently activated upon infection with *L. pneumophila *in T cells, are in agreement with those published by several groups who have also reported *L. pneumophila*-dependent activation of these MAPKs in macrophages and lung epithelial cells [35-38]. However, p38 and JNK activation is flagellin-independent in macrophages [26]. *Legionella *deficient in the Dot/Icm system failed to activate p38 and JNK in macrophages [26,38]. In lung epithelial cells, deletion of the Dot/Icm did not alter IL-8 production, whereas lack of flagellin reduced IL-8 release by *Legionella*, although flagellin- and Dot/Icm-dependency of MAPKs activation was not analyzed [35]. It is likely that *L. pneumophila *flagellin provides signals to T cells as in lung epithelial cells since the *flaA *mutant failed to activate MAPKs in T cells. While it is clear from this report that blockade of p38 with specific inhibitors but not that of ERK, diminishes IL-8 mRNA expression and release in lung epithelial cells [35], the precise molecular mechanism underlying these inhibitions is not clear yet.

We identified both NF-κB and AP-1 binding sites on the 5' flanking region of the IL-8 promoter required for maximal induction of IL-8 by *L. pneumophila*. Because we showed that *L. pneumophila *activated all three MAPKs, we also examined whether *L. pneumophila *triggers MAPKs-mediated IL-8 production via activation of c-Jun, JunD, CREB, and ATF1, which can bind to the AP-1 region in the IL-8 promoter, as well as its cell specificity. By using specific kinase inhibitors, we also demonstrated that IL-8 expression and production in Jurkat cells was sensitive to inhibition of p38 and JNK but not ERK. Consistent with these findings, *L. pneumophila *stimulated phosphorylation of c-Jun, CREB, and ATF1 was blocked by inhibitors of p38 and JNK but not ERK. Using dominant negative mutant proteins of p38α and p38β, we showed that *L. pneumophila *induction of IL-8 was also dependent on the p38 pathway. JunD phosphorylation can be mediated through JNK and ERK pathways [17]. Although both of these molecules were activated in response to *L. pneumophila*, inhibition of JNK and ERK did not reduce phosphorylation of JunD. Further studies are needed to determine the exact kinase responsible for JunD activation.

Overexpression of dominant negative mutants of MyD88 and TAK1 inhibited *L. pneumophila*-induced IL-8 activation. Although we did not examine the effects of these dominant negative mutants on NF-κB and MAPKs activation, our results suggest that trifurcation of *L. pneumophila*-induced IKK-IκB, p38, and MKK4-JNK signaling pathways occurs at TAK1 (Fig. 12).

**Figure 12:** **Schematic representation of *L. pneumophila*-induced signal transduction pathways involved in IL-8 expression human T cells**. The contributions of TLR5 and MKK3/6 are deduced.

## Conclusions

In summary, we showed that *L. pneumophila *induced IL-8 expression and subsequent production through flagellin in human T cells. In addition, the study shed new light on the signaling pathways utilized by *L. pneumophila *in the induction of IL-8. Our findings support the role of IKK-IκB, p38, and JNK signaling pathways in *L. pneumophila *induction of IL-8 in human T cells. Future studies should examine these signaling pathways in T cells of animals and patients infected with *L. pneumophila*, and, if the pathways are found to be significant, a targeted investigation of the role they play in host defense against *L. pneumophila *in infected animals should be performed.

## Methods

### Antibodies and reagents

Rabbit polyclonal antibodies to IκBα and NF-κB subunits p50, p65, c-Rel, p52, and RelB, AP-1 subunits c-Fos, FosB, Fra-1, Fra-2, c-Jun, JunB, and JunD, ATF/CREB family ATF1, ATF2, ATF3, ATF4, and CREB, mouse monoclonal antibody to p52, and goat polyclonal antibody to Lamin B were purchased from Santa Cruz Biotechnology (Santa Cruz, CA). Mouse monoclonal antibody to actin was purchased from NeoMarkers (Fremont, CA). Mouse monoclonal antibody to phospho-IκBα (Ser-32 and Ser-36), rabbit polyclonal antibodies to p65, IKKβ, p38, phospho-p38 (Thr-180 and Tyr-182), MKK4, phospho-MKK4 (Thr-261), phospho-MAPKAPK-2 (Thr-334), phospho-MSK1 (Ser-360), phospho-JNK (Thr-183 and Tyr-185), phospho-c-Jun (Ser-73), and TAK1, and rabbit monoclonal antibodies to phospho-TAK1 (Thr-184 and Thr-187), phospho-IKKβ (Ser-180), CREB, phospho-CREB (Ser-133), ERK1/2, and phospho-ERK1/2 (Thr-202 and Tyr-204) were purchased from Cell Signaling Technology (Beverly, MA). Rabbit polyclonal antibody to phospho-p65 (Ser-536) was purchased from Applied Biological Materials (Richmond, Canada). Bay 11-7082 was purchased from Calbiochem (La Jolla, CA), respectively. p38 MAPK inhibitor SB203580, JNK inhibitor SP600125, and MEK1/2 inhibitor PD98059 were obtained from Sigma-Aldrich (St. Louis, MO).

### Bacterial strains

*L. pneumophila *serogroup 1 strain AA100jm [39] is a spontaneous streptomycin-resistant mutant of strain 130b, which is virulent in guinea pigs, macrophages, and amoebae. The avirulent *dotO *mutant was constructed by random transposon mutagenesis, as described previously [39]. This mutation results in severe defects in intracellular growth and evasion of the endocytic pathway [40]. The Corby *flaA *mutant derived from the wild-type Corby is defective in flagellin [41]. *L. pneumophila *strains were grown at 35°C in a humidified incubator on either buffered charcoal-yeast extract-agar medium supplemented with α-ketoglutarate (BCYE-α) or in buffered yeast extract broth supplemented with α-ketoglutarate (BYE-α). The *flaA *mutant was grown in an environment similar to those used for other strains, but in the presence of 20 μg/ml kanamycin. Heat-killed bacteria were prepared by heating the bacterial suspension at 56°C for 30 min or at 100°C for 1 h. Bacterial inactivation was achieved by treatment with paraformaldehyde (4%, 15 min followed by three washes in phosphate-buffered saline; PBS). Both types of treated suspensions were confirmed to contain no viable bacteria by plating them on BCYE-α agar.

### Cell culture

Human T cells (Jurkat) were maintained in RPMI 1640 medium containing 10% fetal bovine serum (FBS), 100 U/ml penicillin G, and 100 μg/ml streptomycin. Human peripheral blood mononuclear cells (PBMC) were isolated from peripheral blood of healthy donors using Ficoll-Hypaque gradients. PBMC were then further purified using positive selection with immunomagnetic beads specific for CD4 (Miltenyi Biotec, Auburn, CA). On the day of the experiment, cells were refed with fresh antibiotic-free medium and cocultured with *L. pneumophila *for the time intervals indicated below.

### Infection of T cells and intracellular growth kinetics experiments

Jurkat or CD4^+ ^T cells seeded in plates were inoculated with either AA100jm or *dotO *mutant and either Corby or *flaA *mutant at an MOI of 100. In some experiments, heat-killed or paraformaldehyde-fixed bacteria were inoculated in the same manner. At 2 h after infection, cells were centrifuged and the supernatant was discarded. Cells were washed three times with PBS and resuspended in fresh RPMI 1640 medium containing 100 μg/ml gentamycin for 2 h. The cells were washed three times again with PBS and were further incubated with fresh medium. The infected cells and supernatant in each well were harvested at the indicated time intervals by washing the wells three times with sterilized distilled water. These bacterial suspensions were diluted in sterilized water and plated in known volume onto BCYE-α agar. The numbers of CFU in infected cells were counted at the indicated time points after infection.

### Direct fluorescent antibody staining

Jurkat cells were infected with bacteria for 2 h, followed by washing three times with PBS and 2 h gentamycin treatment (100 μg/ml). The infected cells were cultured in fresh antibiotics-free RPMI 1640 medium for an additional 24 h. After being harvested, the cells were fixed in 4% paraformaldehyde for 15 min. Fixed cells were washed with PBS and permeabilized with PBS containing 0.1% saponine and 1% bovine serum albumin for 45 min at room temperature. Permeabilized cells were washed and stained with fluorescein-conjugated mouse anti-*L. pneumophila *monoclonal antibody (PRO-LAB, Weston, FL) for 45 min at room temperature. Finally, the cells were washed and observed under a confocal laser scanning microscope (Leica, Wetzlar, Germany). Cells were stained with the nucleic acid dye 4',6-diamidino-2-phenylindole (DAPI).

### RT-PCR

Total cellular RNA was extracted with Trizol (Invitrogen, Carlsbad, CA) according to the protocol provided by the manufacturer. First-strand cDNA was synthesized from 1 μg total cellular RNA using an RNA PCR kit (Takara Bio Inc., Otsu, Japan) with random primers. Thereafter, cDNA was amplified using 30, 35, and 28 cycles for IL-8, TLRs, and for β-actin, respectively. The specific primers used were as follows: IL-8, forward primer 5'-ATGACTTCCAAGCTGGCCGTG -3' and reverse primer 5'-TTATGAATTCTCAGCCCTCTTCAAAAACTTCTC-3'; TLR2, forward primer 5'-GCCAAAGTCTTGATTGATTGG-3' and reverse primer 5'-TTGAAGTTCTCCAGCTCCTG-3'; TLR3, forward primer 5'-AAGTTGGGCAAGAACTCACAGG-3' and reverse primer 5'-GTGTTTCCAGAGCCGTGCTAA-3'; TLR4, forward primer 5'-TGGATACGTTTCCTTATAAG-3' and reverse primer 5'-GAAATGGAGGCACCCCTTC-3'; TLR5, forward primer 5'-CCTCATGACCATCCTCACAGTCAC-3'and reverse primer 5'-GGCTTCAAGGCACCAGCCATCTC-3'; and for β-actin, forward primer 5'-GTGGGGCGCCCCAGGCACCA-3' and reverse primer 5'-CTCCTTAATGTCACGCACGATTTC-3'. The product sizes were 300 bp for IL-8, 347 bp for TLR2, 320 bp for TLR3, 506 bp for TLR4, 355 bp for TLR5, and 548 bp for β-actin. The thermocycling conditions for the targets were as follows: denaturing at 94°C for 30 s for IL-8, TLR5, and β-actin, and for 60 s for TLR3, and 95°C for 40 s for TLR2 and TLR4, annealing at 60°C for 30 s for IL-8 and β-actin, and for 60 s for TLR3, and 54°C for 40 s for TLR2 and TLR4, and 55°C for 30 s for TLR5, and extension at 72°C for 90 s for IL-8 and β-actin, and for 60 s for TLR2, TLR3, TLR4, and TLR5. The PCR products were fractionated on 2% agarose gels and visualized by ethidium bromide staining.

### Plasmids

The IκBαΔN dominant negative mutant is IκBα deletion mutant lacking the NH_2_-terminal 36 amino acids [11]. The dominant negative mutants of IKKα, IKKα (K44M), IKKβ, IKKβ (K44A), IKKγ, IKKγ (1-305), NIK, NIK (KK429/430AA), MyD88, MyD88 (152-296), and TAK1, TAK1 (K63W), and the dominant negative mutant of either p38α or p38β, have been described previously [19,20,42-44]. Plasmids containing serial deletions of the 5'-flanking region of the IL-8 gene linked to luciferase expression vectors were constructed from a firefly luciferase expression vector [45]. Site-directed mutagenesis of the IL-8 AP-1, NF-IL-6, and NF-κB sites in the -133-luc plasmid was introduced, converting the AP-1 site TGACTCA (-126 to -120 bp) to TatCTCA, the NF-IL-6 site CAGTTGCAAATCGT (-94 to -81 bp) to agcTTGCAAATCGT, and the NF-κB site GGAATTTCCT (-80 to -71 bp) to taAcTTTCCT (lower case letters indicate location of base changes). These constructs were designated as AP-1 site-mutated, NF-IL-6 site-mutated, and NF-κB site-mutated plasmids, respectively.

### Transfection and luciferase assay

Jurkat cells were transfected with 1 μg of the appropriate reporter and 4 μg of effector plasmids using electroporation. After 24 h, *L. pneumophila *was infected and incubated for 6 h. The ratio of bacteria to cells (MOI) was 100. The cells were washed in PBS and lysed in reporter lysis buffer (Promega, Madison, WI). Lysates were assayed for reporter gene activity with the dual luciferase assay system (Promega). Luciferase activity was normalized relative to the *Renilla *luciferase activity from phRL-TK.

### Preparation of nuclear extracts and EMSA

Cell pellets were swirled to a loose suspension and treated with lysis buffer (0.2 ml, containing 10 mM HEPES, pH 7.9, 10 mM KCl, 0.1 mM EDTA, 0.1 mM EGTA, 2 mM AEBSF, and 1 mM DTT) with gentle mixing at 4°C. After 10 min, NP40 was added to a final concentration of 0.6% and the solution was immediately centrifuged for 5 min at 1,000 rpm at 4°C. The supernatants were removed carefully and the nuclear pellets were diluted immediately by the addition of lysis buffer without NP40 (1 ml). The nuclei were then recovered by centrifugation for 5 min at 1,000 rpm at 4°C. Finally, the remaining pellets were suspended on ice in the following extraction buffer (20 mM HEPES, pH 7.9, 0.4 M NaCl, 1 mM EDTA, 1 mM EGTA, 1 mM DTT, 2 mM AEBSF, 33 μg/ml aprotinin, 10 μg/ml leupeptin, 10 μg/ml E-64, and 10 μg/ml pepstatin A) for 30 min to obtain the nuclear fraction. All fractions were cleared by centrifugation for 15 min at 15,000 rpm. NF-κB and AP-1 binding activities with the NF-κB and AP-1 elements were examined by EMSA as described previously [46]. To examine the specificity of the NF-κB and AP-1 element probes, we preincubated unlabeled competitor oligonucleotides with nuclear extracts for 15 min before incubation with probes. The probes or competitors used were prepared by annealing the sense and antisense synthetic oligonucleotides as follows: for the NF-κB element of the IL-8 gene, 5'-GATCCGT**GGAATTTCCT**CTG-3'; for the NF-κB element of the IL-2Rα gene, 5'-GATCCGGCAG**GGGAATCTCC**CTCTC-3'; for the AP-1 element of the IL-8 gene, 5'-GATCGTGA**TGACTCA**GGTT-3', and for the consensus sequence of the CRE, 5'- GATCGATCTTTACCA**TGACGTCA**ATTTGAT-3'. The oligonucleotide 5'-GATCTGTCGA**ATGCAAAT**CACTAGAA-3', containing the consensus sequence of the octamer binding motif, was used to identify specific binding of transcription factor Oct-1. The above bold sequences are the NF-κB, AP-1, CREB, and Oct-1 binding sites, respectively. To identify NF-κB and AP-1 proteins in the DNA-protein complex shown by EMSA, we used antibodies specific for various NF-κB family proteins, including p50, p65, c-Rel, p52, and RelB, various AP-1 family proteins, including c-Fos, FosB, Fra-1, Fra-2, c-Jun, JunB, and JunD, and various ATF/CREB family proteins, including ATF1, ATF2, ATF3, ATF4, and CREB, to elicit a supershift DNA-protein complex formation. These antibodies were incubated with the nuclear extracts for 45 min at room temperature before incubation with radiolabeled probe.

### Western blot analysis

Cells were lysed in a buffer containing 62.5 mM Tris-HCl (pH 6.8), 2% sodium dodecyl sulfate, 10% glycerol, 6% 2-mercaptoethanol, and 0.01% bromophenol blue. Equal amounts of protein (20 μg) were subjected to electrophoresis on sodium dodecyl sulfate-polyacrylamide gels, followed by transfer to a polyvinylidene difluoride membrane and sequential probing with the specific antibodies. The bands were visualized with an enhanced chemiluminescence kit (Amersham Biosciences, Piscataway, NJ).

### Measurement of IL-8

The IL-8 contents in the serum from peripheral blood and the culture supernatants were measured by ELISA (Biosource International, Camarillo, CA). Serum was obtained from healthy volunteers or each patient with *Legionella *pneumonia at diagnosis and stored at -80°C until use. Jurkat and CD4^+ ^T cells were cultured in RPMI 1640 supplemented with 10% FBS in 6-well plates. Cells were infected with *L. pneumophila *for the indicated time intervals. The supernatants were then collected after centrifugation and stored at -80°C until assayed for IL-8 by ELISA. The concentrations of IL-8 were determined using a standard curve constructed with recombinant IL-8. This study was approved by the Institutional Review Board (IRB) of the University of the Ryukyus with license number H20-12-3. Informed consent was obtained from all blood donors according to the Helsinki Declaration.

### Statistical analysis

Values were expressed as mean ± standard deviations (SD). Differences between groups were examined for statistical significance using the Student *t *test. A *P *value less than 0.05 was considered statistically significant.

## Authors' contributions

RT designed and performed the research, analyzed data, and wrote the manuscript. HT participated in the design of the study, performed the research, and analyzed data. ET and CI contributed to the experimental concept and provided technical support. KM, NMu, and JDL carried out the generation of plasmids. KH, FH, and JF provided bacterial strains. NMo established the research plan, supervised the project, and helped to draft the manuscript. All authors read and approved the data and final version of the manuscript.
